The article "Application of Multispectral Imaging in the Human Tympanic Membrane" was published in 2020. Journal: J Healthc Eng.

# Application of Multispectral Imaging in the Human Tympanic Membrane

**DOI:** 10.1155/2020/6219845

**Published:** 2020-09-14

**Authors:** Tien Tran Van, Mi Lu Thi Thao, Linh Bui Mai Quynh, Cat Phan Ngoc Khuong, Linh Huynh Quang

**Affiliations:** ^1^Ho Chi Minh City University of Technology, Faculty of Applied Science, Department of Applied Physics, 268 Ly Thuong Kiet Street, District 10, Ho Chi Minh City 700 000, Vietnam; ^2^National Key Laboratory of Digital Control and System Engineering, 268 Ly Thuong Kiet Street, District 10, Ho Chi Minh City 700 000, Vietnam

## Abstract

Multispectral imaging has recently shown good performance in determining information about physiology, morphology, and composition of tissue. In the endoscopy field, many researches have shown the ability to apply multispectral or narrow-band images in surveying vascular structure based on the interaction of light wavelength with tissue composition. However, there has been no mention to assess the contrast between other components in the middle ear such as the tympanic membrane, malleus, and the surrounding area. Using CT, OCT, or ODT can clearly describe the tympanic membrane structure; nevertheless, these approaches are expensive, more complex, and time-consuming and are not suitable for most common middle ear diagnoses. Here, we show the potential of using the multispectral imaging technique to enhance the contrast of the tympanic membrane compared to the surrounding tissue. The optical absorption and scattering of biological tissues constituents are not the same at different wavelengths. In this pilot study, multiwavelength images of the tympanic membrane were captured by using the otoscope with LED light source at three distinct spectral regions: 450 nm, 530 nm, and 630 nm. Subsequently, analyses of the intensity images as well as the histogram of these images point out that the 630 nm illumination image features an evident contrast in the intensity of the tympanic membrane and malleus compared to the surrounding area. Analysis of such images could facilitate the boundary determination and segmentation of the tympanic membrane (TM) with high precision.

## 1. Introduction

Nowadays, multispectral imaging (MSI) techniques have more and more applications in medical and surgical diagnostics. A multispectral image is a collection of several monochrome images on the same object within specific wavelength ranges. The absorption and reflection of each tissue type are not the same at different wavelengths, and the interaction of light with tissue will fully describe the characteristics of tissue. In the field of dermatology, MSI in visible spectrum has been used to map the distribution of hemoglobin and melanin in skin surface [1, 2] and detect skin cancer lesions [3]. In many other fields, such as gastroenterology and gynecology, MSI techniques have also achieved promising results in tissue observation and become a new diagnosis tool to identify human diseases [4, 5].

The article "Application of Multispectral Imaging in the Human Tympanic Membrane" was published in 2020. Journal: J Healthc Eng.

In human ear, the application of MSI was first studied by Valdez et al. Photos of TM and its surrounding region were taken with otomicroscopy using multichannel LED light source [6]. This result showed that combining blue with green or white light offered much better details of the blood vessel's pattern [6]. In addition, they also proposed that the images taken under red and near-infrared light illumination can be used for detection of pus and infected fluid which accumulate in otitis media [6, 7], in which middle ear infections, also called otitis media, is one of the most common inflammations in children, caused by infection of ear tissue, including the TM and tissues behind it [8]. To diagnose otitis media, most physicians observe blood vessel distribution in the TM as well as the changes of the TM (color, location, mobility of the TM) by using otoscope or endoscopy with white light source. However, determining the changing of TM is not easy for the younger children with the smaller and narrower canals and acute otitis media is the most common in this age group. The early detection and treatment of otitis media can prevent two major problems of complications (such as meningitis, ear infection, and bone necrosis) and hearing loss [8]. Moreover, accurate determination of the TM is also important in case of cochlear implant surgery [9, 10].

Accurate determination of the TM is necessary for correct diagnosis of otitis media. Recently, some researches have developed more algorithms for evaluation or segmentation of TM using endoscope images [11–13]. The first mentioned research is the study of Xie et al. [11]; they used a geometric snake to detect abnormalities in otoscope images. Although this method detected the defects successfully, the elimination of glare might cause the malleus to be lost while it is an important component of the TM. Kuruvilla et al. have developed an algorithm to diagnose the otitis media relying on the TM changes of color, position, and translucence with an accuracy of 89.9% after comparing with the physicians [12]. On the other hand, machine-learning method is also increasingly used in diagnosis of middle ear diseases [14, 15]. Seok et al. show that it is difficult to delineate the exact boundary of the TM; accuracy of TM detection was only 80% when an intersection over union (IoU) score of greater than 0.8 was used [14]. Başaran et al. also used the CNN model and recognized the TM with an average precision of 75.85% [15]. These studies almost used ear endoscopy with white light illumination; however, there are some challenges in brightness and contrast as the lighting, which led to irregularly light fields, and the low contrast of the boundaries in anatomical structures makes automatically structural recognition or segmentation difficult [11–15].

The article "Application of Multispectral Imaging in the Human Tympanic Membrane" was published in 2020. Journal: J Healthc Eng.

In this study, a traditional endoscope was used to capture the images of the reflection of light from the eardrum. Light source was upgraded to high luminance multispectral LEDs with three distinct spectral regions, blue light (450 nm), green light (530 nm), and red light (630 nm), and cold white light (∼6000 K). The absorption properties and depth penetration capacity of different wavelengths in each type of tissue allowed us to improve flexibly images specific for TM, malleus, or blood vessel. Similar approaches have been reported [6]; however, they used otoscope and focused on enhancing the contrast of blood vessels using blue and green spectrum. Here, we focus on the analysis of the image of eardrum captured under red light. Then, the multispectral imaging of human TM was processed by active contour algorithms built on Matlab platform to detect the TM. The segmentation result was analyzed by ENT experts and evaluated by reliable parameters (the Dice similarity coefficient and the Hausdorff distance value).

## 2. Materials and Methods

### 2.1. Optical System Description

A traditional optical endoscope was upgraded with multiwavelength LED light source (see Figure 1). First, endoscope LED RGB light source (Cree manufacturer) with light intensity can be adjusted with a control switch. Next, a fiber optic cable with 2.5 mm diameter and 230 cm long and a rigid endoscope (Provix, Korea) with 2.7 mm diameter and 110 mm long were used to lead the light. To connect the rigid endoscope and camera, an optical C mount coupler for endoscope camera adapter focal length F20 is used. A color CCD camera (Edmund Optics) with a resolution of 976 × 494 pixels is chosen to capture the images and a computer is used for storage and image processing.

### 2.2. Volunteers

The study was approved by the Institutional Evaluation Council of Vietnam National University, Ho Chi Minh City, and conducted according to the principles of the Helsinki Declaration. During the study, we conducted data collection from 12 volunteers, aged 19 to 22 years; the percentage of men and women is equal (Table 1). The middle ear images were taken on both sides of the ear and did not appear to be pathological. Of these 12 sets of images, 7 sets contain blood vessels and the remaining 5 sets have no presence of blood vessels on the tympanic membrane. In Figure 2, a case of normal eardrum was captured using white light. The TM is primarily conical in shape with the apex forming an umbo. The pars flaccida can be identified above the short process of the malleus, and the pars of tensa locate around the umbo. The cone of light region is the reflection of the light used for examining the ear canal, which appears in the anterior-inferior quadrant near the umbo. Blood vessels appear in the wall of meatus as well as in the malleus.

The article "Application of Multispectral Imaging in the Human Tympanic Membrane" was published in 2020. Journal: J Healthc Eng.

### 2.3. Image Segmentation

To segment the TM out of ear canal, active contour algorithm developed by Lankton and Tannenbaum [16] was used. Active contours or snakes are curves and used to define an image domain that can move when it is affected by internal forces coming from the curve itself and external forces computed from the image data. The internal and external forces are defined, so that the snake will conform to an object boundary or other desired features within an image. According to the study of Lankton and Tannenbaum [16], computing these local energies is done with the evolving curve for splitting local neighborhoods into local interior and local exterior. An image is defined on the domain Ω, and let *C* be a closed contour represented as the zero-level set of a signed distance function *φ*. The interior of *C* is specified by the following approximation of the smoothed Heaviside function:

(1) $$\begin{array}{c} ℋ\varphi \left(x\right)=\left\{\begin{array}{cc} 1, & \varphi \left(x\right)<-\varepsilon ,\\ 0, & \varphi \left(x\right)>\varepsilon ,\\ \frac{1}{2}\left\{1+\frac{\varphi }{\varepsilon }+\frac{1}{\pi }\sin\left(\frac{\pi \varphi \left(x\right)}{\varepsilon }\right)\right\}, & \text{otherwise.} \end{array}\right. \end{array}$$

Similarly, the exterior of *C* is defined as (1 − ℋ*φ*(*x*)).

To specify the area just around the curve, we will use the derivative of ℋ*φ*(*x*), a smoothed version of the Dirac delta:

(2) $$\begin{array}{c} \delta \varphi \left(x\right)=\left\{\begin{array}{cc} 1, & \varphi \left(x\right)=\varepsilon ,\\ 0, & \left|\varphi \left(x\right)\right|<\varepsilon ,\\ \frac{1}{2\varepsilon }\left\{1+\cos\left(\frac{\pi \varphi \left(x\right)}{\varepsilon }\right)\right\}, & \text{otherwise.} \end{array}\right. \end{array}$$

To determine the accuracy of the segmentation, the algorithm results will be compared to the ground truth by parameters as the Dice similarity coefficient and the Hausdorff distance value.

The Dice similarity coefficient (DSC) described by Zou et al. [17] is used to measure the overlap segmented TM region between the algorithm and the ground truth detected by ENT specialist. The value is determined by the following formula:

(3) $$\begin{array}{c} \text{Dice}=\frac{2\left|A\cap B\right|}{\left|A\right|+\left|B\right|}. \end{array}$$

Here, *A* is the result zoned by algorithm and *B* is the result zoned by expert otoscopists. The DSC value ranges from 0 to 1. A higher DSC value means that the greater the overlap between the two regions, the more reliable the results.

The article "Application of Multispectral Imaging in the Human Tympanic Membrane" was published in 2020. Journal: J Healthc Eng.

The maximum HD (the Hausdorff distance) is the maximum distance between one point of set *A* and the nearest point of set *B* and defined by [18]

(4) $$\begin{array}{c} HD\left(A,B\right)=\max\left(h\left(A,B\right),h\left(B,A\right)\right), \end{array}$$

(5) $$\begin{array}{c} h\left(A,B\right)=\underset{a\in A}{\max}\underset{b\in B}{\min}a-b. \end{array}$$

‖·‖ is the Euclidean distance between *a* and *b* that are two points on the boundary of set *A* and set *B*.

## 3. Results and Discussion

A case of a normal tympanic membrane is illustrated in Figure 3. The images are captured using white light illumination (a), red light (b), green light (c), and blue light (d). By direct observation only, it is difficult to distinguish some differences in monocolor image. So these color images (Figures 3(a)–3(d)) were converted into the grayscale images corresponding to Figures 3(e)–3(h). The image obtained using the white light (see Figures 3(a) and 3(e)) have ear details including malleus handle, blood vessels, incus, and cone of light. On the theory of optical absorption, hemoglobin has high absorption in the blue and green regions of the spectrum; therefore, using green and blue light illumination offered much better details of the blood vessels. White light LED has also two regions of spectrum: one narrow peak at blue region and another wide peak at green-yellow region. In our system, the vascularity can be observed clearly in the white and green images. The image with blue light affords the lack of illumination in ear cavity which caused identifying poorly the characterization of the TM and blood vessels. This is also leading to create a false boundary and the unsmooth border (see Figure 3(h)).

Our interest here focuses on the absorption in the red light region of the TM and tissues surrounding. First, in the visible spectrum, hemoglobin has the lowest absorption in the region of red light; therefore, the blood vessels did not appear in the red image (see Figures 3(b) and 3(f)). Second, the absorption of collagen is higher than hemoglobin in the red light spectrum [19]. The TM is a thin membrane tissue, consisting of three types of collagen, I, II, and III [20]. Particularly, the middle layers of the pars tensa and annulus are very rich in collagen fibers [21]. Some researchers have shown that red image can be used to express absolute appearance of melanin on the skin [1] or collagen on the breast [19]. Therefore, red image could also be used to produce a high contrast image for collagen structures in the TM. Last, red light penetrates deeper into the tissue than blue and green light. For all of these reasons, the red image has many advantages like increased accuracy of structural identification and functional assessment of the tympanic membrane. The optical characteristic of each tissue type is not the same under different illumination conditions. For more clearly direct observation of the structure of the middle ear, we provide the jet colormap (J) of the multispectral images shown in Figure 3, which is the J white image (a), the J red image (b), the J green image (c), and the J blue image (d) in Figures 4(a)–4(d), respectively. We can see that the distribution of colorscale values on the J white image and the J green image is quite the same; both inside and outside of the tympanic membrane have multiple color levels indicated in Figures 4(a) and 4(c). The J blue image (see Figure 4(d)) is illuminated by a low light source with lots of noise and cannot provide accurate information about the boundary of the tympanic membrane. Interestingly, in the J red image (see Figure 4(b)), there is a significant difference between TM region and the outside of TM region. The handle of malleus appears in the same color as outside of TM. In particular, the outside skin region of the eardrum is relatively homogeneous in component and color and unaffected by noise as other images. Thence, it is possible to distinguish the boundaries of the eardrum and the surrounding area better than the rest of the images.

The article "Application of Multispectral Imaging in the Human Tympanic Membrane" was published in 2020. Journal: J Healthc Eng.

Next, we offer the region histogram and the line histogram as an evidence to assess the feasibility of detecting TM. First, Figures 4(e)–4(h) show the region histogram maps of the middle ear corresponding to Figures 4(a)–4(d), in which the mean values of TM and wall of meatus (outside of TM) have been measured inside and outside of the ellipse curve as shown in Figure 4(a). A mean value of handle malleus has been measured inside rectangle as shown in Figure 4(b). When superimposing the histograms of J white image and J green image for the TM region and the outside of TM region (wall of meatus), the overlap of two peaks is observed, as shown in Figures 4(e) and 4(g)). The histogram of J blue image also has two very large peaks because of the noise (Figure 4(h)). This is the main reason leading to the inability to segment the TM includes the malleus using threshold-based algorithms. On the other hand, in the region histogram of J red image as shown in Figure 4(f), the overlap of histogram for the inside and outside TM of this image is less than the J white image, J green image, and J blue image. The overlap between the charts is due to the malleus and the wall of the meatus having the same intensity value. The histogram of the outside TM of the J red image has a narrow peak with the homogeneous intensity distribution as can be seen in Figure 4(f). Based on the above results, it is proved that the multispectral imaging can be used to analyze tissue properties of human middle ear and the red image is best suited for identification and segmentation of TM in the middle ear.

In addition, we also provide the line histogram with two special lines (see Figure 4(a)), the first line through the handle of malleus called horizontal line and the second line which is perpendicular to the first line and through the cone of light called vertical line. The intersection of each line (A-A′ and B-B′) and ellipse will provide the information of the intensity at the boundary between the TM and the surrounding area. As we can see, the line profiles of Figures 5(a)–5(d) show the strong variation of the intensity at the left boundary and the less change at the right boundary (marked by red dots). This is caused by the malleus attached to the TM, from umbo to the wall of meatus. Besides, the line profiles of Figures 5(e)–5(h) also have strong intensity variations at the upper as well as the under boundary of eardrum (marked by red dots). It proves that using the active contour algorithm is very suitable for the segmentation of the eardrum in this case.

Based on the endoscope device, we proceed to collect 12 series of data of normal TM from volunteers. Each set has four images captured with white, red, green, and blue light and they are completely similar in both size and position of features on the TM. To ensure the stable segmentation result, we choose the white image for putting an ellipse mask which covered the TM and the ground truth was defined by expert endoscopists.  Figure 6 shows a set of representative images of normal TM. The results of segmentation algorithm are shown in Figures 6(a)–6(d). Figures 6(e)–6(h) indicate the comparison of the ground truth and segmentation results shown in pairs. We found that the result of segmentation of TM includes malleus in the red image which is better than the other images because it has the closest border with the doctor's result and the contour of the red image is smoother than the others. To demonstrate that results are reliable, the need for a method could accurately evaluate the segmentation results of TM. The suitable parameters are the DSC value and the maximum HD.

The article "Application of Multispectral Imaging in the Human Tympanic Membrane" was published in 2020. Journal: J Healthc Eng.

Firstly, the DSC could compute the ratio of overlap between the segmentation result by using algorithm and the ground truth defined by the endoscopy experts. However, the active contour algorithm based on different images gives completely different results in shape as well as boundary size with the same mask and number of loops. The eardrum segmentation results in white and green images (Figures 6(e) and 6(g)) are significantly different from ground truth, although the DSC index is quite high on four different wavelength images. The boundary in the white and green images has a part protruded and recessed in the pars flaccida leading to the fact that the border is not smoothed, while the DSC value computed based on the number of pixels coincided between the segmentation result and the ground truth. Thus, we require another standard parameter which could measure the coincidences of the segmentation results compared with the ground truth and the maximum HD (the Hausdorff distance) is one of the appropriate options.

The DSC (see Figure 7(a)) and the maximum HD (see Figure 7(b)) diagrams are the average value of the segmentation results in 12 series of images showing the difference of four different wavelengths. Generally, in the DSC chart, the red images group have the highest accurate average value of about 0.91 (higher DSC value is good). In contrast, in the maximum HD chart, the red images group have the lowest average value of about 9.00 in length unit (lower max HD value is good) that demonstrated the consistency of the TM segmentation results. The obtained results showed a good result when using active contour on red image to segment the TM which include malleus, with the highest DSC value and the lowest maximum HD value.

## 4. Conclusions

Endoscopy is a standard method for diagnosing ear disease, combined with a multispectral light source that can provide more information about the pathology and morphology of the middle ear. We modified the multispectral LED light source based on two maximum absorption peaks and one minimum absorption peak of the hemoglobin corresponding to the blue, green, and red spectrum. The study results indicated that the red illumination image not only fully described the contrast enhancement of the tympanic membrane and malleus compared to the surrounding tissue but also minimized the noise appearing on the image. We demonstrate the efficacy of this research in an TM segmentation application with high accuracy. Determining exactly the position as well as the boundary of TM helps to evaluate middle ear disease faster and better. Increasing the middle ear components contrast, especially the TM and malleus, does not only improve the ability to observe directly the morphological structure tympanic membrane in some cases of inflammation, redness, and vascular proliferation but also support the preprocessing step in biomedical image analysis researches.

The article "Application of Multispectral Imaging in the Human Tympanic Membrane" was published in 2020. Journal: J Healthc Eng.

## Figures and Tables

**Figure 1:** The endoscope model: LS: LED light source and control; R: rigid endoscope; CM: optical C mount coupler; CCD: Color CCD camera; FO: fiber optic cable.

**Figure 2:** The white image of normal right eardrum was captured using endoscope. 1: TM (orange circle). 2: handle of malleus. 3: pars flaccida. 4: pars of tensa. 5: umbo. 6: cone of light. 7: blood vessel. 8: wall of meatus.

**Figure 3:** A normal right eardrum: (a) white image, (b) red image, (c) green image, (d) blue image, and (e–h) grayscale images of (a), (b), (c), and (d). (a) White image. (b) Red image. (c) Green image. (d) Blue image. (e) White grayscale image. (f) Red grayscale image. (g) Green grayscale image. (h) Blue grayscale image.

**Figure 4:** Comparison of intensity images and region histograms obtained with the multispectral imaging on the tympanic membrane shown in Figure 3. (a–d) show the intensity image of white, red, green, and blue image. (e–h) show the region histograms of J white, J red, J green, and J blue image, respectively.

**Figure 5:** Comparison of the line histogram corresponding to the J white, J red, J green, and J blue image shown in Figure 4. (a–d) the horizontal histogram; (e–h) the vertical histogram.

**Figure 6:** Results of segmentation of the tympanic membrane: (a, e) white, (b, f) red, (c, g) green, and (d, h) blue. Green color is the results of algorithm, pink color is ground truth, and white color is the overlapping.

**Figure 7:** Average metric values of segmentation results of tympanic membrane: (a) Dice value and (b) max HD.

**Table 1:** Summary of data collection.

Sample	Age (years)	Pathology	Blood vessel	Image(s)
7	19–22	Normal	✓	28
5	19–22	Normal	✕	20

## Data Availability

In this study, 12 volunteers with 48 images of the tympanic membrane, accepted by the ethics committees of Vietnam National University, Ho Chi Minh City, Vietnam from 2019, were used as study objects. The authors cannot share it or make it available online for privacy reasons.
